# Anchor-Free Braille Character Detection Based on Edge Feature in Natural Scene Images

**DOI:** 10.1155/2022/7201775

**Published:** 2022-08-08

**Authors:** Liqiong Lu, Dong Wu, Jianfang Xiong, Zhou Liang, Faliang Huang

**Affiliations:** ^1^Guangdong Provincial Key Laboratory of Development and Education for Special Needs Children, Lingnan Normal University, Zhanjiang 524048, China; ^2^School of Computer Science and Intelligence Education, Lingnan Normal University, Zhanjiang 524048, China; ^3^School of Computer and Information Engineering, Nanning Normal University, Nanning 530001, China

## Abstract

Braille character detection helps communication between normal and visually impaired people. The existing Braille detection methods are all aimed at scanning Braille document images while ignoring natural scene Braille images and CNN shining in the field of pattern recognition is rarely used for Braille detection. Firstly, a natural scene Braille image data set named NSBD was constructed. Then, an anchor-free Braille character detection based on the edge feature was proposed by analyzing that Braille characters in natural scene images that are relatively small in size, and a Braille character is composed of Braille dots that werelocated at the edge region of Braille character. Finally, the performance of the proposed method and other classic methods based on CNN was compared on NSBD. The experimental results show that the proposed method has good performance.

## 1. Introduction

There are about 17 million visually impaired people in China, and one visually impaired person is born every minute [1]. Braille is an important way for these people to learn knowledge and communicate with other normal people. But, for normal people, such as the parents, teachers, and friends of these visually impaired people, it is very difficult to know well about Braille and then leads to insurmountable obstacles when communicating with visually impaired people. Braille recognition aims to help normal people and visually impaired people to communicate without barriers, such as teachers checking the students' homework rapidly and parents viewing the students' dairy to know more about them. Braille character detection is an important prestep for Braille recognition.

Braille text consists of Braille characters, and each character is a rectangular block called a Braille cell. A Braille cell contains six Braille dots arranged in three rows and two columns with 64 different combinations [2]. In previous work, Braille detection methods often aimed at scanned document images. In these methods, Braille dots were first detected; then the detected dots were combined into Braille characters for recognition [2–4]. Actually, firstly, it is difficult to scan Braille texts anytime and anywhere. With the development of society, it has become very convenient to take out a mobile phone to take pictures of Braille texts at any time. Therefore, Braille recognition in natural scene images becomes a more mainstream application scenario. Secondly, it needs to combine several Braille dots with a Braille character for Braille recognition. This multistep operation may accumulate more errors, thereby reducing the performance of Braille recognition. Based on the above analysis, we studied Braille character detection in natural scene images as shown in Figure 1. Firstly, a natural Braille image data set named NSBD was constructed. Then CNN shining in the field of pattern recognition [5–9] was introduced, and an anchor-free Braille character detection method based on edge feature was proposed. Finally, the performance of the proposed method and other classic methods was compared on NSBD. The comparison results show that the proposed method can detect Braille characters effectively in natural scene Braille images.

The rest of this paper is organized as follows. In Section 2, we briefly introduce some related work. Our proposed database and approach are described in Sections 3 and 4, respectively.  Section 5 presents the experimental results, and finally, Section 6 summarizes the paper.

## 2. Literature Review

We review the related literature from the following two aspects: the work of public Braille image data sets and the work of Braille detection methods.

Currently, there are very few public data sets on Braille detection and recognition. Existing Braille detection methods are tested on their small-scale data sets with different acquisition ways [10–13]. Li et al. constructed a public Braille document image data set named DSBI that consists of 114 double-sided Braille images from 6 Braille books and some ordinary printed documents divided into 26 images for train and 88 images for test [3]. The Braille document images in DSBI are all acquired by the flat-bed scanner, so all Braille texts are carefully aligned. The annotation is made by specifying the rotation angle, the coordinates of each row and column after rotation, and whether there is a Braille character in each row and column. DSBI is the first public Braille document image, and its research significance is self-evident. While in the real world, it is very difficult to scan Braille documents to images anytime, anywhere. Nowadays, people can use a mobile phone to get images easily. So we constructed a natural scene Braille image data set named NSBD in which all Braille images are captured by mobile phone or downloaded from the Internet. We believe that the construction of the natural scene Braille image data set conforms to the real application scene and is conducive to the communication between visual impaired people and normal people.

Braille is only used by special populations, so there is a little research on Braille detection. Previous work on Braille detection mainly focused on Braille text in documents. Since Braille text in document has cells of a fixed size, and the arrangement of Braille rows and columns is fixed, most of the previous methods detect Braille dots first, and then combined Braille dots to obtain Braille characters. These Braille dots detection methods can be divided into two types. One is based on image segmentation. Another is to first mine Braille features and then to use some machine methods to detect Braille dots.

Image-segmentation-based methods usually firstly used a local adaptive thresholding method to segment the Braille image into several parts such as shadows, light, and background then identified Braille recto and verso dots through the combination rules of these parts [10–14]. This type of Braille dots detection method was sensitive to the thresholding value and getting the final result through multiple steps was easy to accumulate errors. In order to avoid the above problems, another type of Braille dot detection method directly detected Braille dots by combining manual feature mining and machine learning methods. Features and machine learning methods include Haar and SVM [3]; HOG and SVM [15]; Haar, LBP, HOG, and Adaboost [16]; and others. Morgavi et al. used a simple neural network to detect Braille dots [17]. Venugopal-Wairagade used Hough transform for circle detection to find Braille dots [18].

In recent years, methods for directly detecting Braille characters have begun to appear. Li et al. used a segmentation CNN with modified UNet [19] architecture to detect Braille characters directly at CVPRW 2020 [20]. In this work, they used a neural network to determine which pixels belong to Braille characters, and then subsequent postprocessing was required to aggregate multiple pixels to form Braille characters based on the segmentation results. Actually, as the most effective technology in the field of object detection [21–23], CNN is rarely applied to the field of Braille detection. We think there is more work to do for the research of Braille character detection based on CNN.

Summarizing the work on Braille detection, it is found that the following two problems have not been solved well. The first is that there are few public Braille image data sets, especially a lack of natural scene image data sets. Another is that most Braille dots detection methods detect Braille characters in multiple steps, which tends to accumulate errors. And there are few works for Braille character detection based on CNN. Based on the above analysis, we constructed a natural Braille image data set and used CNN to propose an anchor-free Braille character detection method based on edge features. We also compared the performance between our method and other classic methods.

## 3. NSBD: Natural Scene Braille Image Data Set

We constructed a natural scene Braille image data set named NSBD. Different from the existing Braille image data set, all Braille images in NSBD are natural scene images and are obtained in two ways. Some images are downloaded from the Internet, and the other images are taken with mobile phones. There are a total of 212 images in NSBD where 164 images are used for training and others are used for testing.

### 3.1. Braille Images in NSBD

Unlike Braille characters in scanned Braille document images, which have a simple and uniform background, consistent size, and regular arrangement. Braille characters in natural scene images have different backgrounds, different size, different colors, and so on. Especially, some Braille characters in images are blurry and blend with the background, making them extremely difficult to detect, as shown in Figure 2. In Figure 2, Braille characters in natural scenes exist on a variety of backgrounds including walls, cards, and elevator buttons; the size of Braille characters varies greatly; the color and direction of Braille characters are also different. These characteristics of Braille characters in natural scene images make them difficult to be detected by the existing methods proposed for scanned Braille document images.

In addition, there are some Braille document images taken with a mobile phone. These images are skewed at different angles, and the lights shining on the Braille character are not uniform; Braille characters and Chinese characters are mixed together as shown in Figure 3.

### 3.2. Label Files in NSBD

Braille characters in all images in NSBD are marked with rectangle boxes. We used the tool named Labelme to mark all Braille characters and then used the generated JSON files to generate label files in VOC format and ICDAR format with MATLAB code. The structure of the database folder is shown in Figure 4. There are three folders that represent the original image and label files, ICDAR format files, and VOC format files. In the original files, each Braille image corresponds to two files: JSON file and txt file. Each line in the txt file represents the position of a Braille character (coordinate values of the upper left and lower right corners). In ICDAR format files, each Braille image corresponds to a txt file. Each line in the txt file represents the coordinate values of four vertices in the clockwise direction. In VOC format files, each Braille image corresponds to a xml file in which the coordinate values of the upper left and lower right vertices of all Braille character rectangles are given.

## 4. Methods

We firstly analyzed the characteristics of Braille characters in natural scene images and the structure difference between Braille characters and Chinese and English characters. Then we combined the edge feature of Braille character and the idea of the anchor-free method, a classic object detection technology suitable for small object detection in CNN, to propose an anchor-free Braille character detection method based on edge feature in natural scene images.

### 4.1. Characteristics of Braille Characters in Natural Scene Images

As shown in Figure 5, Braille characters in natural scene images are always small and vary in size, color, and background. Especially, some Braille characters are blended with the background. As the most effective tool for mining object features in natural scene images in recent years, CNN has achieved excellent performance. So we think CNN is a good choice to mine the features of Braille characters in natural scene images. In addition, activated by the work in [24], we analyze that Braille characters in natural scene images are relatively small in size and are suitable to use the anchor-free method for detection.

We further analyze the difference in writing between Braille characters and common characters such as Chinese or English characters. Chinese or English characters consist of strokes, and these strokes fill the middle region of characters. While Braille characters consist of Braille dots, and these Braille dots are located at the edges, not the middle region of the Braille character rectangle as shown in Figure 6. So we think the pixels at the edge of the Braille character are the key to Braille character detection.

We concluded that Braille characters in natural scene images have the main following characteristics: (1) in addition to the inherent characteristics of text in natural scene images, Braille characters in natural scene images are mostly small in size. (2) Braille characters consist of Braille dots that are discontinuous and only located at the edge of Braille characters. Based on the above analysis, we proposed an anchor-free Braille character detection method based on edge features. In our method, firstly ResNet-50 [25] was used as the backbone of CNN, and different size feature layers were merged to mine the Braille character feature fully. Then Braille character pixels at the edge were detected on a larger feature map. Finally, the distances of these pixels to the four sides of the character rectangle were predicted. We will introduce our proposed method below from the framework of our approach, the loss function, and how to predict Braille character rectangle.

### 4.2. The Framework of Our Approach

The framework illustration of our approach is shown in Figure 7. We selected ResNet-50 as the backbone of CNN. There are five stages of feature maps with different sizes in ResNet-50, and these feature maps are merged to mine the features of Braille characters according to formula (1). In formula (1), *f*_*i*_ is the feature map of the *i*-th layer in ResNet-50, and *h*_*i*_ is the merged feature map of *h*_*i-1*_ and *f*_*i*_. Considering that the Braille character is relatively small, we finally perform the prediction of edge line map and geometry map at the feature map whose size is (*H/2* × *W/2*). Here, *H* and *W* are the height and width of the input image, respectively.

(1) $$\begin{array}{c} \left\{\begin{array}{c} h_{1}=f_{1},\\ h_{i+1}={\text{conv}}_{3\times 3}\left({\text{conv}}_{1\times 1}\left(\text{Concat}\left(f_{i+1},{\text{Unpooling}}_{2\times 2}\left(h_{i}\right)\right)\right)\right),\;i=1,2,3,4,\\ h_{5}={\text{conv}}_{3\times 3}\left(h_{5}\right). \end{array}\right) \end{array}$$

The edge line map and the geometry map are the geometric presentation of the Braille character rectangle. In our approach, the edge line map is designed to find the pixels at the edge region, and the geometry map is designed to get the distance from each pixel located at the edges to the four sides of the Braille character rectangle.  Figure 8 gives the Braille character rectangle, edge region, and the distance from a pixel located at the edge region to the four sides of the Braille character rectangle.

Here, we take the left 1/3 region and the right 1/3 region as the edge region. For one pixel in the input image, if this pixel is in the edge region, its label is 1 else 0. We use *d*_1_, *d*_2_, *d*_3_, and *d*_4_ to represent the distance from one pixel located at the edge region to four sides of the Braille character rectangle. For a pixel *P* (*x, y*), the coordinates of the upper left and lower right corners of its corresponding Braille character rectangle are (*x*_*ul*_, *y*_*ul*_) and (*x*_*lr*_, *y*_*lr*_), respectively. If equation (2) is satisfied, this pixel is in the edge region. Equation (3) is utilized to calculate the value of *d*_1_, *d*_2_, *d*_3_, and *d*_4_.

(2) $$\begin{array}{c} x-x_{ul}\leq \frac{x_{lr}-x_{ul}}{3},\\ \text{or }x-x_{ul}\geq \frac{2*\left(x_{lr}-x_{ul}\right)}{3}, \end{array}$$

(3) $$\begin{array}{c} d_{1}=x-x_{ul},\\ \;d_{2}=x_{lr}-x,\\ d_{3}=y-y_{ul},\\ d_{4}=y_{lr}-y. \end{array}$$

### 4.3. Loss Function

For pixel detection at the edge region and distance prediction from each pixel to four sides of the Braille character rectangle, we designed the corresponding loss function. Equation (4) gives the total loss function that consists of the above two parts, and the parameter *α* is utilized to set the weight of Loss_edge_. Like EAST, the value of *α* is set to 0.01. Equation (5) gives the calculation method of *Loss* geometry. In equation (5), *N* is the total number of pixels located at the edge region; *A*^*i*^_*inter*_ represents the intersection area of a ground-truth rectangle and predicted rectangle; and *A*^*i*^_*union*_ represents the union area of a ground-truth rectangle and predicted rectangle. Equations (6) and (7) give the calculation of *A*^*i*^_*nter*_ and *A*^*i*^_*union*_. In equations (6) and (7), *d*_1g_, *d*_2g_, *d*_3g_, and *d*_4g_ and *d*_1*p*_, *d*_2*p*_, *d*_3*p*_, and *d*_4*p*_, respectively, represent the ground-truth distances and predicted distances from a certain pixel to the four sides of the Braille character rectangle. We use the dice coefficient [26] to calculate Loss_edge_. In equation (8), *T*_edge_ and *P*_edge_ represent the ground-truth edge region matrix and the predicted edge region matrix, respectively.

(4) $$\begin{array}{c} \text{Loss}={\text{Loss}}_{\text{geometry}}+\;\alpha \times {\text{Loss}}_{\text{edge}}, \end{array}$$

(5) $$\begin{array}{c} {\text{Loss}}_{\text{geometry}}=\frac{1}{N}\sum_{i=1}^{N}\left(-\log\frac{A_{\text{inter}}^{i}+1}{A_{\text{union}}^{i}+1}\right), \end{array}$$

(6) $$\begin{array}{c} A_{\text{inter}}=\left(\min\right.\left(d_{1g},\;d_{1p}\right)+\min\left(d_{3g},\;d_{3p}\right)*\;\left(\min\left(d_{2g},\;d_{2p}\right)+\min\left(d_{4g},\;d_{4p}\right)\right), \end{array}$$

(7) $$\begin{array}{c} A_{\text{union}}=\left(d_{1p}+d_{3p}\right)*\left(d_{2p}+d_{4p}\right)+\left(d_{1g}+d_{3g}\right)*\left(d_{2g}+d_{4g}\right)-A_{\text{inter }}, \end{array}$$

(8) $$\begin{array}{c} {\text{Loss}}_{\text{edge}}=1-\frac{2*\sum \left(T_{\text{edge}}*P_{\text{edge}}\right)}{\sum T_{\text{edge}}*T_{\text{edge}}+\sum P_{\text{edge}}*P_{\text{edge}}}. \end{array}$$

### 4.4. Predicting Braille Character Rectangle

In the testing stage, taking an image containing Braille characters as input, the trained CNN model outputs an edge region matrix, and lots of distance values predicted by pixels located at the edge region. Algorithm 1 is used to predict the Braille character rectangle.

Firstly, only pixels with a value greater than or equal to 0.8 are considered valid pixels; then four distances predicted by these valid pixels are used to get Braille character rectangles according to equation (9). In equation (9), (*x, y*) is the coordinate value of a valid pixel, and (*y*_*ul*_*, y*_*ul*_) and (*x*_*lr*_*, y*_*lr*_) are, respectively, the coordinates of the upper left and lower right pixel of the Braille character rectangle predicted by this pixel.

(9) $$\begin{array}{c} x_{ul}=x-d_{1},\\ y_{ul}=y-d_{3},\\ x_{lr}=x+d_{2},\\ y_{lr}=y+d_{4}. \end{array}$$

After the above steps, many Braille character rectangles with the overlapping area are obtained. How to choose and get the best prediction results is the next problem to be solved. NMS [27] is a good choice to handle this situation, but NMS uses a pairwise comparison, which runs in O (*n*^2^) and *n* is the number of pixels at the edge region of the Braille character rectangle. EAST proposed Locality-Aware NMS that runs in O (*n*) in best scenarios. We analyzed that our method only uses pixels at the edge of the Braille character rectangle, and these pixels are distributed in the vertical direction. So we modified the row-by-row merging in Locality-Aware NMS to column-by-column merging, and for a column, only the last merged one was retained. This improved technique conforms to the characteristics of Braille character and is more efficient.

## 5. Results

We have used the open-source Tensorflow [28] framework to run on commercial GPUs using GTX 2080. During the training phase, all CNNs used in this method are optimized by stochastic gradient descent (SGD). We set the initial learning rate 10^−4^, and the change process of the learning rate adopts the same exponential decrease as EAST. The maximum number of training was set to 100,000. We also compared the detection performance of our proposed Braille character detection approach with other methods on two data sets named NSBD and DSBI.

### 5.1. Evaluation Protocol of Braille Character Detection

We used the classical evaluation protocol for text detection that relies on precision (*P*), recall (*R*), and *H*mean to evaluate the performance of our approach. Precision represents the proportion of correctly detected Braille characters among all detected Braille characters. If the IOU between the predicted rectangle and the ground-truth rectangle is greater than 0.5, the prediction is considered correct. The recall is used to evaluate whether all Braille characters are all detected. *H*mean is a composite indicator determined by the values of precision and recall. Generally, *H*mean is used to evaluate the quality of a detection algorithm, and the larger this value is, the better the detection performance of the algorithm. Equation (10) lists the calculation process of these three indicators. *TP* is the number of correctly detected Braille characters, and *FP* is the number of wrongly detected Braille characters. *FN* is the number of Braille characters that are not detected by the method.

(10) $$\begin{array}{c} P=\;\frac{TP}{FP+TP},\\ R=\frac{TP}{TP+FN\;}\text{,}\\ H\text{ mean}=2\times \frac{P\times R}{P+R}. \end{array}$$

### 5.2. Braille Character Detection Performance on NSBD

We have compared the detection performance between our approach and other classic object detection methods including faster RCNN, SSD, and EAST. As shown in Table 1, compared with other methods, our approach achieved the best Braille character detection performance. The values of recall and *H*mean are 0.555 and 0.689, respectively.

Compared with faster RCNN and SSD, our method achieved the best detection performance in precision, recall, and *H*mean. Compared with EAST, our method has an obvious advantage in recall, which increases recall from 0.462 to 0.555. EAST and our method are all based on an anchor-free framework. As an excellent text detection method, EAST first detects the pixels in the central region and then detects their corresponding text rectangle. We analyzed the difference between Braille characters and Chinese and English characters and then proposed the idea of first detecting the pixels in the edge region and then detecting their corresponding Braille character rectangle. Viewing the experimental results, this idea is correct and valid. Our method can indeed detect more Braille characters in natural scene images.Bold font indicates maximum value.

We also used different structures of CNN in our method for Braille character detection. ResNet-50 and VGG-16, the classic CNN structures, were all used in our method, and the detection results were compared. As shown in Table 2, our method using VGG-16 as the basic CNN structure achieved the value of precision and recall, respectively, of 0.908 and 0.549. Although this detection performance is slightly lower than the detection performance achieved by our method using ResNet-50 as the basic CNN structure, it obviously surpassed the detection performance achieved by SSD, Faster RCNN, and EAST.

### 5.3. Braille Character Detection Performance on DSBI

We also compared the performance of our method with other existing methods on DSBI where all images are acquired by the flat-bed scanner. Braille characters in scanned document images are densely arranged, having a small fixed size and a simple background. Since the features of Braille characters in scanned document images are very different from those in natural scene images, when verifying on the DBSI data set, we simplified our method. Firstly, we detected the edge regions of Braille characters and then merged the two adjacent edge regions into a rectangular Braille character box. Finally, Braille characters that are too big or too small were filtered out.

The detection performance of our method and others on DSBI has been listed in Table 2. Our method achieved the value of *H*mean of 0.977 that is 0.02 less than the optimal value achieved by BraUNet [20]. Although our method has not achieved the best performance, as a Braille character detection method designed in natural scene images, our method can also detect Braille characters in scanned document images effectively.

### 5.4. The Analysis of Braille Character Detection Samples

We have listed the detection correct samples and partially correct samples, respectively, in Figures 9 and 10. Our approach can detect correctly all Braille characters of different sizes, colors, and writing styles in a variety of images with different backgrounds as shown in Figure 9. We also listed some image samples in which a small number of Braille characters are not detected by our approach in Figure 10. When Braille characters in images are particularly dense, with uneven lighting or shadows, our method did not detect all Braille characters, but the detected Braille characters have high accuracy. In the future, we will focus on the above situations and improve our method to detect more Braille characters.

## 6. Conclusions

The field of Braille recognition lacks public data sets especially for natural scene images and Braille character detection methods based on CNN are rarely studied. So we constructed a natural scene data set named NSBD. Then we analyzed that Braille characters in natural scene images are always small in size and Braille characters consist of Braille dots located at the edge. Finally, we proposed an Anchor-free Braille character detection method based on edge features in natural scene images.

In our method, ResNet-50 was used as the backbone of CNN, and different size feature layers were merged to mine the Braille character feature fully. Then Braille character pixels at the edge region were detected on a larger feature map. Finally, the distances of these pixels to the four sides of the character rectangle were predicted. Our method achieved the detection performance with a precision of 0.910 and *H*mean of 0.689 on NSBD that are better than the detection performance of classic object detection methods such as SSD, faster RCNN, and EAST. But, our method only detects partly Braille characters when Braille characters in images are particularly dense, with uneven lighting or shadows.

In the future, we will continue our work from the following two aspects. Firstly, we will focus on the work of how to detect more Braille characters in the above situations. We initially consider introducing a multidimensional attention mechanism and combing coarse detection and fine detection to improve the detection performance of Braille characters. The attention mechanism helps efficiently mine the position of Braille edge points, and the combination of coarse detection and fine detection can better detect Braille characters of different sizes. Secondly, we will use the LSTM network and the correspondence between Braille and Chinese to translate the detected Braille characters into Chinese characters.

## Figures and Tables

**Figure 1:** Braille character detection in a natural scene image.

**Figure 2:** Natural scene Braille images.

**Figure 3:** Braille document images taken by mobile phone.

**Figure 4:** The structure of the database folder. Images and label files have been shared, and the corresponding network link is https://pan.baidu.com/s/10WqYvC3BDltl6cTTwtUEmQ?pwd=499i.

**Figure 5:** Braille characters in natural scene images are small and vary in size, color, and background.

**Figure 6:** (a) Braille characters, (b) Chinese characters, and (c) English characters.

**Figure 7:** The framework illustration of our approach.

**Figure 8:** Braille character rectangle, edge region, and the distance from a pixel located at the edge region to the four sides of the Braille character rectangle.

**Figure 9:** Detecting correctly samples with our method.

**Figure 10:** Detecting partly correct samples with our method.

**Algorithm 1:** The process of predicting Braille character rectangles.

**Table 1:** Comparison of experimental results on NSBD.

Method	P	R	*H*mean
SSD [17]	0.809	0.545	0.651
Faster RCNN [18]	0.790	0.502	0.614
EAST [19]	**0.930**	0.462	0.616
Our method (ResNet-50)	0.910	**0.555**	**0.689**
Our method (VGG-16)	0.908	0.549	0.684

**Table 2:** Comparison of experimental results on DSBI.

Method	P	R	*H*mean
BraUNet [20]	**0.9935**	0.9988	**0.9966**
UNet [20]	0.9828	0.9669	0.9751
TS-OBR [20]	0.9928	**0.9996**	0.9962
Our method	0.9581	0.9981	0.977

Bold font indicates maximum value.

## Data Availability

The data used to support the results of our study are public on the network, and the link is https://pan.baidu.com/s/10WqYvC3BDltl6cTTwtUEmQ?pwd=499i.
